This article has been retracted.

# Risk Factors of Catheter-Related Infection in Unplanned Extubation of Totally Implantable Venous-Accessportsin Tumor Patients

**DOI:** 10.1155/2022/4235316

**Published:** 2022-09-27

**Authors:** Min Xu, Lie Deng, Yanyi Zhu, Yuanfang Li, Fan Wang, Hui Li, Ying Zhou

**Affiliations:** ^1^Breast Surgery Affiliated Cancer Hospital, Institute of Guangzhou Medical University, Guangzhou 510000, China; ^2^Radiotherapy Area 5, Affiliated Cancer Hospital, Institute of Guangzhou Medical University, Guangzhou 510000, China; ^3^Nursing Department Affiliated Cancer Hospital, Institute of Guangzhou Medical University, Guangzhou 510000, China

## Abstract

**Background:**

Totally implantable intravenous ports (TIVAPs) are mostly used for long-term intravenous infusion therapy in cancer patients and can be left in the body for long periods of time for easy management, making them a simple and safe infusion device. Although the risks associated with long-term retention of fully implantable IV ports are less than those associated with other intravenous catheters, various complications may still occur at the time of implantation or during long-term use.

**Purpose:**

To provide a scientific basis for clinical reduction of implantable intravenous port-associated infection complications by studying the risk factors for catheter-associated infection complications in patients applying implantable intravenous ports.

**Methods:**

A retrospective study was conducted on oncology patients treated with TIVAP at our hospital between January 2017 and November 2021, with a review of patients who were unplanned for extubation. Their demographic data, underlying disease status, and surgery-related data were counted to summarize and analyze the complications and related influencing factors of implantation and postimplantation.

**Results:**

A total of 70 individuals with a mean age of 56.49 ± 12.19 years were included in the study. Among them, 39 were male and 64 had the highest percentage of epithelial tumors, followed by tumors of the lymphopoiesis system and mesenchymal tumors with 4 and 2 cases, respectively. Forty-eight of these patients did not have their ports removed as planned due to the occurrence of catheter-related hematogenous infections. In univariate analysis, BMI and neutropenia were risk factors for catheter-associated infections. In the multivariate analysis, BMI (OR = 1.38, 95% CI: 1.07–1.78, *p*=0.013) was an independent risk factor for catheter-associated infections.

**Conclusions:**

The overall complication rate of fully implanted intravenous ports was high, but most complications improved with symptomatic management, and no deaths due to port complications were identified. Infection was the most common complication, with catheter-associated bloodstream infection being the most common cause of unplanned port extraction. Patients with a higher BMI were at high risk of developing implantable IV port-associated infections, which may be an independent risk factor for implantable IV port-associated infections.

## 1. Introduction

According to the data released by China's tumor registry in 2012, the incidence and mortality of tumors in China have been increasing at an accelerated rate, with about 3.5 million new cancer cases and 2.5 million deaths due to cancer each year [1, 2]. Malignant tumors not only seriously threaten the life safety of patients but also bring a heavy economic burden and great psychological pressure to patients' families, while the long treatment period of malignant tumors and the frequent need for repeated chemotherapy bring serious inconvenience and disturbance to patients' life. Patients with malignant tumors, especially those with advanced malignant tumors, need to rely on intravenous supply for various therapeutic drugs and nutrition, and repeated venipuncture can bring a series of side effects such as damage to the venous wall; meanwhile, chemotherapy drugs and hypertonic drugs can easily cause phlebitis, and if the operation is not proper, once the chemotherapy drugs leak out, it may cause local tissue necrosis and increase patients' pain. Therefore, it is especially important to establish a long-term, safe, and convenient infusion channel.

Since its clinical application, intravenous catheterization has shown its advantages in several ways, especially in obese, edematous, and cachectic patients, and in patients where superficial veins are difficult to find, it is extremely important to establish reliable deep venous access. Most of the central venous catheters terminate at the junction of the superior vena cava and right atrium, thus, during drug infusion, irritating drugs such as hypertonic drugs and chemotherapeutic drugs can be rapidly diluted by a high flow rate and high flow of blood, rapidly reducing the damage of irritating drugs to the vessel wall. When intravenous cannulation is applied to tumor patients as the route of infusion of irritant drugs and chemotherapy drugs, it obviously solves the damage of irritant drugs and chemotherapy drugs to peripheral veins and at the same time provides a good way for patients' treatment. There are 3 major types of central venous catheter placement techniques commonly used in clinical practice, namely: central venous catheter (CVC), peripherally inserted central catheter (PICC), and implantable venous access port (IVAP). [3, 4]. The disadvantages of peripherally inserted central catheters and IVAPs have been reported in the literature because a portion of the catheter interface is exposed to the body surface, increasing the risk of catheter-related infections and interfering with patients' daily activities [5, 6].

The implantable intravenous port, also known as the implantable central venous port access system (CVPAS), is a deep vein placement technique, the most important feature of which is that it can be implanted subcutaneously for long-term retention in the body [7]. It establishes an ideal long-term intravenous access, consisting of an injection seat for puncture and an intravenous catheter system, suitable for infusion of chemotherapy drugs, hypertonic drugs, parenteral nutrition fluids, and blood products, as well as for blood sample collection, among others. IV access is established by simply puncturing the noninvasive needle vertically through the base of the infusion port, which reduces the pain caused to the patient by repeated punctures of the peripheral veins while protecting the vessels. Since its first application by Chang et al. in 1983 [8], it has been gradually promoted for its convenience of portability, simplicity of daily care, low maintenance cost, reduction of the number of punctured vessels, improvement of patients' quality of life, and long service life, and is adapted to patients requiring long-term, repeated intravenous infusion therapy and chemotherapy. In China, the implantable intravenous infusion port technology was introduced in 1988 and was first reported in 1998 [9], and with the promotion of the use of the IVAP technology and the growth of patient demand, this technology was gradually accepted and applied in many hospitals in China. The occurrence of IVAP-related complications not only prolongs patients' hospital stays and shortens the use of infusion ports, but also increases the economic burden on patients. Therefore, it is important to understand and be familiar with IVAP-related complications in order to prevent, detect, and manage them in a timely manner.

Complications of IVAP are classified as early and late complications. Early complications refer to complications that occur during the period from intraoperative or postimplantation to the first use of the implantable IVAP, which mainly include vascular and nerve injury, hematoma formation, hemothorax, hemopneumothorax, air embolism, pericardial tamponade, arrhythmia, etc.; late complications refer to complications that occur after the first use of the implantable IVAP, which mainly include catheter-related infections, thrombosis, catheter occlusion, and cardiac arrhythmia. It mainly includes catheter-related infections, thrombosis, catheter occlusion, drug extravasation, catheter displacement or fracture, catheter entrapment syndrome, superior vena cava ulceration or perforation, and infusion seat overturning [10, 11], and catheter-related infections are the most common among them. Studies [12, 13] reported that 46.2% of patients who had their infusion port removed during use did so because of catheter-associated infections, a rate much higher than complications such as thrombosis or other dysfunctions. According to relevant data, despite the fact that infusion ports reduce the chance of bacterial infection, 3–10% of infusion ports are removed once complications of infusion port-associated infections occur [14]. A study [15] analyzed complications associated with IVAP treatment and found that IVAP-associated bacteremia was the most expensive to treat. Risk factors for IVAP complications have been reported differently in the literature and include operative technique, patient age, gender, choice of puncture route, type of tumor (parenchymal organ tumor, hematologic tumor), the patient's own physical condition, type of chemotherapeutic agent, and IVAP-related care. It has been reported in the literature [16] that malignant hematologic disease is the most significant risk factor for catheter-associated infections. Studies [17] have found that catheter-associated infections are common in young patients with the malignant hematologic disease, and it has been hypothesized that this may be due to intense chemotherapy and neutropenia. In contrast, other literature in recent years has reported a lower rate of infection in outpatients using IVAP. In this study, we analyzed which factors increase the occurrence of infectious complications in patients with IVAP to provide some valid and scientific references for reducing the incidence of IVAP infections in future clinical work.

## 2. Methods

### 2.1. Participants

A retrospective survey was conducted of patients who received TIVAP for cancer at our institution between January 2017 and November 2021 and patients who were unplanned for extubation. Approval was obtained from our hospital ethics committee, and informed consent was obtained from each patient.

Inclusion criteria: ① patients with a preliminary clinical diagnosis of malignancy by cytology, histopathology, or bone marrow pathology, or preoperatively by imaging and relevant tumor indicators, and who were clearly diagnosed by pathology after surgery, and who underwent IVAP placement and maintenance in our hospital; ② patients who required long-term and repeated infusion therapy; ③ patients with IVAP implanted through the subclavian and internal jugular veins.

Exclusion criteria: ① combined systemic infection; ② uncontrolled infection in the tissue surrounding the IVAP implantation site; ③ abnormal coagulation function (PLT < 50/nl, PT < 50%, or INR > 1.5); ④ history of acute thrombosis and occlusion of the subclavian and superior vena cava.

### 2.2. Data Collection

The collected data included demographic information (age, sex, BMI, education, smoking, alcohol, surgical history, history of central vein catheterization, comorbidities, medication history, and tumor type), laboratory reports (erythrocytes, leukocytes, platelets, C-reactive, international normalized ratio (INR), activated partial thromboplastin time (APTT), D-Dimer, and neutrophils), and TIVAP-related information (operation duration, postoperative infusion port interval, secondary adjustment of the infusion port position, implantation method, catheter placement site, conduit material, infection occurred ten days after catheterization, iatrogenic skin injury, missing extraction of the infusion needle, irregular catheter care, home catheter, surgery during indwelling TIVAP, radiotherapy at the indwelling site, and catheter retention time). In the present study, the first outcome was TIVAP-related infection. TIVAP-related infection was defined as documented bacteremia and colonization of the catheter tip with the same microorganisms (significant microbial growth), signs of infection (fever, chills, and/or hypotension), and no obvious source of bacteremia other than the catheter [16]. Tumor types are classified as epithelial tumors, lymphopoietic system tumors, and mesenchymal tumors.

### 2.3. TIVAP Procedure

All TIVAP procedures are performed by the surgeon under local anesthesia in the operating room under sterile conditions. The surgical access can be through the subclavian or internal jugular veins on both sides or arm veins on both sides, depending on the patient's vascularity at the puncture site, skin condition, and treatment modality. Internal jugular vein implantation is used as an example. The patient is placed in a supine position with the head tilted back and turned to the opposite side. After routine anesthesia and disinfection, the puncture site is determined, the puncture is performed under ultrasound guidance, and blood is drawn back to determine whether the puncture was successful. After a successful puncture, a guide wire is introduced in the direction of the puncture needle, and the skin and subcutaneous tissue are dilated using a skin dilator, after which a catheter is introduced, a capsule bag is bluntly separated, an infusion port holder is implanted in the capsule bag, the catheter is connected to the syringe, and a noninvasive butterfly needle is used. The injection seat was punctured, and the infusion port and catheter were then checked for patency with sodium heparin saline. Finally, the skin was sutured. After the puncture was completed, the chest X-ray was determined to be free of twisting and knotting of the catheter before use.

### 2.4. Catheter Care

Maintenance care of the CVC was performed by experienced nurses according to Infusion Nursing Standards of Practice, including daily inspection of the skin around the port of infusion for pressure, swelling, hematoma, and infection. The use of 10–20 ml of saline to flush the tube at the beginning and end of the infusion and every 4 h during continuous infusion or between infusions of two drugs with contraindications. At the same time, 3–5 ml of heparin-saline solution at a concentration of 100 *μ*/mL is used to seal the tube under positive pressure at the end of the infusion and after the flush. If the tube is not used for a long time, the CVC will be maintained every 4 weeks, including the flush and seal.

### 2.5. Statistical Analysis

For baseline characteristics, variables were expressed as mean ± standard deviation (SD) or proportions. Differences in baseline characteristics between the catheter-associated infection group and other reason groups were assessed using Student's *t*-tests, the chi-square test for continuous variables, and Fisher's exact test for categorical variables. Risk factors associated with catheter-associated infections were analyzed univariately using logistic regression analysis, and those with *p* values < 0.10 were included in multivariate analysis. The results were expressed as the ratio (OR), with a ratio of 95%.

## 3. Results

### 3.1. Patient Characteristics

A retrospective study of oncology patients treated with TIVAP in our hospital between January 2017 and November 2021 and unplanned extubation was conducted. Their demographic data, underlying disease status, and procedure-related data were counted to summarize and analyze implantation and postimplantation complications and related influencing factors. A total of 70 individuals, with a mean age of 56.49 ± 12.19 years, were finally included in the study. Among them, 39 were male and 64 had the highest percentage of epithelial tumors, followed by tumors of the lymphopoietic system and mesenchymal tumors with 4 and 2 cases, respectively. Forty-eight of these patients did not have their ports removed as planned due to the occurrence of catheter-related hematogenous infections. Forty-eight of these patients had unscheduled port removal due to the occurrence of catheter-associated hematogenous infection, 12 were removed due to catheter obstruction or thrombosis formation, 6 were removed due to port exposure and extravasation, and 4 were removed due to puncture port infection. Catheter-associated bloodstream infections occurred in 48 patients, 23 of whom were male, aged 30–90 years, with a procedure length of 0.5–1.5 hours, a mean catheter retention time of 245.08 ± 418.50 days, and catheter use of mostly 3–7 days per month (Table 1).

### 3.2. Comparison between Catheter-Associated Infections Group and Other Reason Group

The clinical presentation of catheter-associated bloodstream infections often includes chills, fever, chills, or erythema, swelling, and pain at the site of catheter placement, nodules, and/or pus exudation. Because of the lack of specificity and sensitivity, the diagnosis of CRBSI should not be based solely on this basis, and care should be taken to distinguish between catheter-associated bloodstream infections that originate from the catheter and those that arise from other sites because some catheter-associated bloodstream infections are secondary to surgical incisional infections, nosocomial pneumonia, gastrointestinal infections, and urinary tract infections. Therefore, catheter-associated bloodstream infections are only considered to be bloodstream infections caused by catheter infections and can exclude other sources. Also, the culture of the head end of the catheter is the same pathogenic organism as the blood culture, but it is difficult to distinguish between the two in the current clinical practice. In addition, some studies have shown that local inflammatory manifestations are uncommon in the presence of catheter-associated infections, with Gram-positive bacteria being the main pathogenic organism in CRBSI, and it is rare for this organism to cause local or systemic signs of infection. CRBSI should be considered to be caused by an *aureus* or Gram-negative bacillus infection if there is a clear manifestation of inflammation at the placement site along with fever, chills, or obvious clinical signs of systemic infection [18]. In the absence of laboratory results, in patients with clinical manifestations of bloodstream infection such as chills and fever, if the body temperature returns to normal after removal of the suspected catheter, it can only be used as indirect evidence of catheter-associated infection but not definitively as CRBSI. Therefore, when a catheter-associated infection is suspected, catheter specimen culture and blood culture results should be obtained to further clarify the diagnosis.

There were no significant differences between the catheter-associated infections group and the other reason group in terms of age, sex, educational level, tumor classification, surgical history, smoking history, history of central venous catheterization, anticoagulant drug use history, hypertension, diabetes, erythrocyte abnormality, leukocyte abnormality, platelet abnormality, abnormal C-reactive protein, INR abnormality, APTT abnormality, D-Dimer abnormality, operation duration, postoperative infusion port interval, secondary adjustment of infusion port position, implantation method, catheter placement site, conduit material, infection occurred ten days during catheterization, Iatrogenic skin injury, missing extraction of infusion needle, irregular catheter care, home catheter maintenance, surgery during indwelling TIVAP, radiotherapy at the indwelling site, and catheter retention time. Patients with the catheter-associated infections group had a higher BMI (23.55 ± 3.41 vs. 21.74 ± 2.85, *p*=0.034), and a higher rate of neutropenia (45.8% vs. 18.2%, *p*=0.026) than the other reason group (Table 1).

### 3.3. Risk Factors

The risk factors for catheter-related infection in unplanned extubation of totally implantable venous-access ports in tumor patients were reported in Tables 1 and 2. According to the univariable analysis, BMI and neutropenia were risk factors for catheter-related infection. According to the multivariable analysis, BMI (OR = 1.38,95%CI:1.07–1.78, *p*=0.013) was an independent risk factor for catheter-related infection (Table 2).

## 4. Discussion

The purpose of treatment of advanced malignant tumors is usually to reduce 'patients' pain, prolong 'patients' survival, and improve patients' quality of life. Intravenous chemotherapy and nutritional support are one of the important means for the clinical treatment of advanced malignant tumors, and because of long-term repeated infusions of chemotherapy drugs and multiple punctures, patients' extravasation of chemotherapy drugs leads to an increased incidence of peripheral local tissue necrosis and peripheral phlebitis, which seriously affects the treatment of patients and aggravates their pain. The implantable intravenous infusion port began to be used for clinical intravenous infusion in the 1980s [19], and IVAP technology has been successfully applied in recent years for postoperative chemotherapy of malignant tumors such as lung cancer, breast cancer, and cervical cancer and for patients who repeatedly require intravenous infusion multiple times and have difficulty in peripheral infusion, all of which have achieved outstanding results [20]. Implantable intravenous ports have been compared with external infusion devices in much literature, and the conclusions reached are that implantable intravenous ports are relatively less risky. Studies [21] have shown that implantable intravenous ports are better than PICCs in reducing the occurrence of infections in patients with hematologic malignancies, not only by greatly reducing the number of punctured veins but also by smoothly delivering drugs directly to the central vein. Also, it can not only greatly reduce the number of punctured veins, but also smoothly deliver drugs to the central vein, greatly reduce the damage of chemotherapy drugs and hypertonic drugs to peripheral veins, and reduce the occurrence of phlebitis. Studies in the literature [22] have shown that the IVAP technique, as one of the permanent intravenous infusion routes for oncology patients, shows a reduced incidence of infection compared with other infusion techniques and improves the quality of life in patients with malignant tumors.

The TIVAP consists of two parts: an internal catheter and an infusion seat, including a subcutaneous implant port (or reservoir) connected to a central venous catheter, most often inserted into the internal jugular, subclavian, or cephalic veins. As the preferred intravenous access for oncology chemotherapy patients, TIVAP not only reduces the pain associated with repeated punctures but also avoids damage to the peripheral vasculature from highly concentrated and highly irritating chemotherapeutic agents. Also, because the TIVAP load is buried in the body, it has little impact on the patient's image and normal life, resulting in greater patient acceptance and satisfaction. However, factors affecting unplanned TIVAP removal, such as catheter-associated infections, remain a current concern. Therefore, it remains important to explore the risk factors for catheter-associated infections and to investigate how to prevent them. In this study, based on the unplanned extraction population, 48 patients developed catheter-associated bloodstream infections, and the rate of catheter-associated infections was 67.6%, which was much higher than in other studies. The rate of neutropenia in patients in the catheter-associated infection group (45.8% vs. 18.2%, *p*=0.026) was higher than in the other causes group, similar to previous studies that reported that cancer patients are more susceptible to bacterial infections due to immunocompromise [23]. Interestingly, we calculated the interval between postoperative TIVAP use and found no difference in catheter-associated infections caused by TIVAP use within 24 hours versus 24 hours later, implying that delayed postoperative TIVAP use does not increase the incidence of catheter-associated infections. This has some guiding value for the use of clinical TIVAP but, of course, still requires subsequent confirmation with a larger sample size. In addition, we found that BMI was an independent risk factor for catheter-associated infections by multifactor regression analysis. This suggests that the more obese people are, the higher the incidence of catheter-associated infections. This may be because the accumulation of adipocytes promotes inflammation and alters hormonal secretion patterns, and these changes tend to alter the immune system, making obese individuals more susceptible to bacterial infections. In addition, BMI as a risk factor for infection has been demonstrated in other studies [24]. Although BMI cannot be changed to a great extent during hospitalization, early prevention in patients with a higher BMI is of greater clinical importance.

Before considering how to prevent TIVAP catheter-associated infections, it is important to understand the mechanisms of bacterial infection. First, the lack of proper disinfection procedures during TIVAP catheter implantation allows microorganisms to migrate along the catheter surface and is a major cause of catheter-associated infections. Second, inappropriate disinfection measures during TIVAP maintenance can also lead to bacterial infections. In addition, intraluminal infections caused by microbial migration into the catheter lumen are a common route of infection. Another possible but uncommon cause is distant blood-borne bacterial infections. Therefore, prevention of TIVAP catheter-associated infections should begin with insertion, which should be performed with strict sterilization guidelines. In addition, real-time ultrasound-guided intravenous cannulation and proper skin preparation are key to preventing catheter-associated infections. In addition, strict asepsis should be implemented during dressing changes and maintenance. Numerous studies have shown that the use of chlorhexidine gluconate with alcohol disinfection is effective in reducing the rate of catheter microbial colonization [25]. In addition, the skin around the TIVAP should be carefully assessed daily for signs of infection, such as pressure pain and swelling. More importantly, enhanced psychological care and related health education for patients also play an important role in the prevention of TIVAP catheter-associated infections, and we believe that good prevention can effectively reduce the incidence of TIVAP catheter-associated infections.

There are some limitations to this study. First, this study is a single-center retrospective study. Secondly, the sample size of this study was small. However, this study concludes that BMI is an independent risk factor for TIVAP catheter-associated infections and is the first one reported to date, which has some guiding value for clinical practice. This can be validated in subsequent studies using a large sample of data.

## 5. Conclusion

The overall complication rate of fully implanted intravenous ports was high, but most of the complications improved with symptomatic management, and no deaths due to port complications were identified. Infection was the most common complication, with catheter-associated bloodstream infection being the most common cause of unplanned port extraction. BMI (OR = 1.38, 95% CI: 1.07 to 1.78, *p*=0.013) was an independent risk factor for catheter-associated infection. In patients with a higher BMI, we should enhance care to prevent the development of catheter-associated infections.

## Figures and Tables

**Table 1:** Univariate analysis of catheter blood flow infection leading to infusion portpullout.

Characteristics	Catheter-associated infections (*n* = 48)	Other reason (*n* = 22)	*p*
Age (years)	57.65 ± 11.58	53.95 ± 13.36	0.242^a^
Male	23 (47.9%)	16 (72.7%)	0.052^b^
BMI (kg/m^2^)	23.55 ± 3.41	21.74 ± 2.85	**0.034**
Bi index (points)	96.04 ± 15.16	97.27 ± 11.72	0.737
Educational level	—	—	0.454
Primary school and below	18 (37.5%)	5 (22.7%)	—
Middle school	24 (50.0%)	13 (59.1%)	—
University and above	6 (12.5%)	4 (18.2%)	—
Tumor classification	—	—	0.808^b^
Epithelial tumor	20 (90.9%)	44 (91.7%)	—
Lymphohematopoietic system tumor	1 (4.5%)	3 (6.3%)	—
Mesenchymal tumor	1 (4.5%)	1 (2.1%)	—
Surgical history	13 (27.1%)	5 (22.7%)	0.699
Smoking history	16 (33.3%)	8 (36.4%)	0.804
History of central venous catheterization	4 (8.3%)	0 (0%)	0.401
Anticoagulant drug use history	4 (8.3%)	0 (0%)	0.401
Hypertension	13 (27.1%)	2 (9.1%)	0.089
Diabetes	9 (18.8%)	2 (9.1%)	0.303
Erythrocyte abnormality	16 (33.3%)	5 (22.7%)	0.369
Leukocyte abnormality	13 (27.1%)	2 (9.1%)	0.089
Platelet abnormality	13 (27.1%)	3 (13.6%)	0.214
Abnormal C-reactive protein	22 (45.8%)	9 (40.9%)	0.700
INR abnormality	7 (14.6%)	5 (22.7%)	0.401
APTT abnormality	14 (29.2%)	2 (9.1%)	0.063
D-dimer abnormality	15 (31.3%)	11 (50%)	0.132
Neutropenia	22 (45.8%)	4 (18.2%)	**0.026**
Operation duration (h)	0.89 ± 0.27	0.85 ± 0.27	0.616
Postoperative infusion port interval		—	0.916
<24°h	41 (85.4%)	19 (86.4%)	—
≥24°h	7 (14.6%)	3 (13.6%)	—
Secondary adjustment of infusion port position	1 (2.1%)	1 (4.5%)	0.566
Implantation method	—	—	0.329
Ultrasonic guidance	14 (29.2%)	4 (18.2%)	—
Blind puncture	34 (70.8%)	18 (81.8%)	—
Catheter placement site	—	—	0.584
Internal jugular vein	18 (37.5%)	8 (36.4%)	—
Subclavian vein	27 (56.3%)	11 (50.0%)	—
Vein of arm	3 (6.3%)	3 (13.6%)	—
Conduit material	—	—	0.566
Polyurethane	47 (97.9%)	21 (95.5%)	—
Silica gel	1 (2.1%)	1 (4.5%)	—
Infection occurred ten days after catheterization	1 (2.1%)	3 (13.6%)	**0.053**
Iatrogenic skin injury	4 (8.3%)	4 (18.2%)	0.229
Missing extraction of infusion needle	2 (4.2%)	0 (0%)	0.331
Irregular catheter care	7 (14.6%)	2 (9.1%)	0.524
Home catheter maintenance	6 (12.5%)	2 (9.1%)	0.677
Surgery during indwelling TIVAP	4 (8.3%)	2 (9.1%)	0.916
Radiotherapy at the indwelling site	6 (12.5%)	2 (9.1%)	0.677
Catheter retention time (days)	245.08 ± 418.50	127.18 ± 87.70	0.068

^a^ANOVA; ^b^chi square test.

**Table 2:** Analysis of influencing factors for catheter-related blood source infection.

Variable	*B*	*S.E.* (*B*)	Wald	*p*	OR (95%CI)
BMI	0.321	0.129	6.235	**0.013**	1.38 (1.07–1.78)
Catheter retention time (days)	0.001	0.002	0.340	0.560	1.00 (0.99–1.01)
Female	1.175	0.828	2.011	0.156	3.24 (0.64–16.42)
Hypertension	1.619	0.935	3.001	0.083	5.05 (0.81–31.55)
Neutropenia	1.663	0.920	3.263	0.071	5.27 (0.87–32.04)
Infection occurred ten days after catheterization	−3.872	2.024	3.659	**0.056**	0.02 (0–1.10)
Abnormal leukocyte level	1.742	1.282	1.846	0.174	5.71 (0.46–70.48)
APTT level abnormality	1.464	1.311	1.248	0.264	4.32 (0.33–56.42)

## Data Availability

The experimental data used to support the findings of this study are available from the corresponding author upon request.
